The article "Influence of the Level of Emergency Medical Facility on the Short-Term Treatment Results of Cardiac Arrest: Out-of-Hospital Cardiac Arrest and Interhospital Transfer" was published in 2022. Journal: Emerg Med Int.

# Influence of the Level of Emergency Medical Facility on the Short-Term Treatment Results of Cardiac Arrest: Out-of-Hospital Cardiac Arrest and Interhospital Transfer

**DOI:** 10.1155/2022/2662956

**Published:** 2022-08-27

**Authors:** Je Young Chung, Yuri Choi, Jinwoo Jeong, Sung Woo Lee, Kap Su Han, Su Jin Kim, Won Young Kim, Hyunggoo Kang, Eun Seog Hong

**Affiliations:** ^1^Department of Emergency Medicine, Dong-A University Hospital, Busan, Republic of Korea; ^2^Department of Emergency Medicine, Dong-A University College of Medicine, Busan, Republic of Korea; ^3^Department of Emergency Medicine, Korea University College of Medicine, Seoul, Republic of Korea; ^4^Department of Emergency Medicine, Asan Medical Center, University of Ulsan College of Medicine, Seoul, Republic of Korea; ^5^Department of Emergency Medicine, Hanyang University College of Medicine, Seoul, Republic of Korea; ^6^Department of Emergency Medicine, Ulsan University Hospital, University of Ulsan College of Medicine, Ulsan, Republic of Korea

## Abstract

**Objective:**

This study aimed to elucidate whether direct transport of out-of-hospital cardiac arrest (OHCA) patients to higher-level emergency medical centres (EMCs) would result in better survival compared to resuscitation in smaller local emergency departments (EDs) and subsequent transfer.

**Methods:**

This study was a retrospective population-based analysis of cases registered in the national database of 2019. This study investigated the immediate results of cardiopulmonary resuscitation for OHCA compared between EMCs and EDs and the results of therapeutic temperature management (TTM) compared between the patients directly transported from the field and those transferred from other hospitals. In-hospital mortality was compared using multivariate logistic regression.

**Results:**

From the population dataset, 11,493 OHCA patients were extracted. (8,912 in the EMC group vs. 2,581 in the ED group). Multivariate logistic regression revealed that the odds for ED mortality were lower with treatment in EDs than with treatment in EMCs. (odds ratio 0.712 (95% confidence interval (CI): 0.638–0.796)). From the study dataset, 1,798 patients who received TTM were extracted. (1,164 in the direct visit group vs. 634 in the transferred group). Multivariate regression analysis showed that the odds ratio for overall mortality was 1.411 (95% CI: 0.809–2.446) in the transferred group. (*p* = 0.220).

**Conclusion:**

The immediate outcome of OHCA patients who were transported to EDs was not inferior to that of EMCs. Therefore, it would be acceptable to transport OHCA patients to the nearest emergency facilities rather than to the specialized centres in distant areas.

The article "Influence of the Level of Emergency Medical Facility on the Short-Term Treatment Results of Cardiac Arrest: Out-of-Hospital Cardiac Arrest and Interhospital Transfer" was published in 2022. Journal: Emerg Med Int.

## 1. Introduction

Despite global efforts to improve cardiopulmonary resuscitation (CPR) and post-resuscitation management, cardiac arrest remains a major global health problem and a leading cause of mortality [1, 2]. The incidence of out-of-hospital cardiac arrest (OHCA) in the Republic of Korea increased from 19,480 cases in 2006 to 29,832 cases in 2016 [3]. Efforts to improve the prognosis of cardiac arrest patients have been implemented, including the adoption of international guidelines for CPR, training of laypersons for bystander CPR, and implementing standardised training programs for advanced cardiovascular life support (ACLS) by healthcare providers [3–5]. Recently, along with early recognition of arrests and prompt resuscitation, there has been an emphasis on comprehensive post-resuscitation care, including targeted temperature management (TTM) and percutaneous coronary intervention (PCI) [6–8] .The current international guidelines for CPR introduce the concept of a cardiac arrest centre (CAC), where advanced and comprehensive post-resuscitation management is available, and suggest that transporting cardiac arrest patients to the centres would improve survival and neurologic prognosis [9–11]. However, it remains unclear whether transporting cardiac arrest patients directly to these centres from the scene would improve their prognosis as compared to promptly transferring them after the restoration of spontaneous resuscitation (ROSC) at other hospitals. A recent study reported that both cases had favourable outcomes and did not find any evidence that direct transport from the scene would have a superior outcome than that of secondary transfer to the CACs [5].

Not all countries, including Korea, have an emergency medical system (EMS) capable of on-scene ACLS [12, 13]. In these situations, mandatory transport of patients undergoing CPR to advanced centres might delay the initiation of ACLS, thereby impairing the treatment outcomes. However, this would enable the early application of post-resuscitation procedures such as TTM. Moreover, ACLS is a labour-intensive process that imposes a substantial burden on the already overcrowded emergency medical centres (EMCs), while the equipment and skills needed for it are widely available in the emergency departments (EDs) in smaller hospitals. Therefore, it would be worth investigating whether directly transporting cardiac arrest patients to higher-level emergency centres would indeed improve the treatment results, which would guide appropriate field triage and determination of the destination hospital.

This study aimed to elucidate whether direct transport of OHCA patients to higher-level EMCs would result in better survival compared to resuscitation in smaller local EDs and subsequent transfer by analysing the nationally collected and maintained database of emergency medical care usage [14].

The article "Influence of the Level of Emergency Medical Facility on the Short-Term Treatment Results of Cardiac Arrest: Out-of-Hospital Cardiac Arrest and Interhospital Transfer" was published in 2022. Journal: Emerg Med Int.

## 2. Materials and Methods

### 2.1. Study Settings and Design

This study was a retrospective population-based analysis of cases registered in the National Emergency Department Information System (NEDIS) maintained by the National Emergency Medical Center of the Republic of Korea. The NEDIS prospectively collects demographic and clinical data of patients treated in the EDs of all emergency medical facilities in Korea. The National Health Insurance Services (NHIS) covers the entire Korean population and medical institutes; therefore, the NHIS claims database contains all insurance claims, including those for procedures and medications [1]. The claim codes are matched to the corresponding ED visits in the NEDIS dataset using unique identifiers before being anonymised and provided to the researchers.

This study comprised two parts of the investigation. First, the immediate results of CPR for OHCA were compared between higher-level EMCs and local EDs. Second, the results of post-resuscitation management represented by TTM in the EMCs were compared between the patients directly transported from the field and those transferred from other hospitals. Cases eligible for analyses were extracted from the NEDIS dataset, utilising the information on initial evaluation and insurance claims as filters.

The study was reviewed and approved by the Institutional Review Board of the Dong-A University Hospital, and informed consent was waived because the study utilised a de-identified version of the preexisting national dataset (DAUHIRB-EXP-22-023).

## 3. Study Population

Anonymised data regarding consecutive emergency visits between 1 January, 2019, and 31 December, 2019, that were registered in the NEDIS database were provided for this research (reference number: N20211820511).

## 4. Treatment Results of Prehospital Cardiac Arrest Cases

The first part of the study compared the outcomes of CPR in OHCA. The cases that met the following criteria were extracted from the dataset: age ≥15 years; transported to the ED via the National Fire Department ambulance service, which is the mainstay of prehospital care in Korea; heart rate or blood pressure values of 0 or unmeasurable; and insurance claim codes for CPR registered in the ED. Patients presenting with injury or poisoning and those transferred from other hospitals were excluded. Data regarding the level of the emergency medical facility, sex, age, mode of transport to the ED, disposition from the ED, length of stay in the ED, and treatment results after hospital admission were collected. In-hospital mortality between the EMCs and local EDs was compared using multivariate logistic regression.

The article "Influence of the Level of Emergency Medical Facility on the Short-Term Treatment Results of Cardiac Arrest: Out-of-Hospital Cardiac Arrest and Interhospital Transfer" was published in 2022. Journal: Emerg Med Int.

## 5. Outcome of Targeted Temperature Management Conducted in the Emergency Medical Centres

The second part of the study evaluated the treatment outcomes of patients who underwent TTM in EMCs. Because a substantial proportion of cardiac arrest patients resuscitated in local EDs were transferred to other hospitals for advanced care, the outcome of those cases needed to be evaluated. Therefore, we compared the in-hospital mortality of the patients who received TTM in EMCs between those who directly visited the EMCs and those transferred to the EMCs from other hospitals. The data on patients aged ≥15 years and insurance claim codes for TTM registered in the EDs or after admission were extracted from the study population and analysed. Patients with poisoning or injury and those who were alert on arrival to the ED were excluded.

Data on age, sex, level of the emergency medical facility, mode of transport to the ED, consciousness based on the alert, voice, pain, unresponsive scale, initial vital signs on arrival to the ED, disposition from the ED, length of stay in the ED, and treatment results after hospital admission were collected. In-hospital mortality was compared between the direct visit group and the transferred group using multivariate logistic regression. The modified early warning score (MEWS) was calculated based on consciousness and vital signs and was incorporated into the regression model instead of individual variables to ensure a linear correlation with mortality and to avoid multicollinearity problems.

## 6. Statistical Analysis

Statistical analyses were conducted using *R* 4.1.1 (R Foundation for Statistical Computing, Vienna, Austria, 2021). Categorical variables are presented as counts and percentages and continuous variables are presented as mean and standard deviations. The categorical variables were compared using the chi-square test and the continuous variables were compared using independent *t* tests. Multivariate logistic regression was used to compare the ED mortality or the in-hospital mortality between the groups after adjusting for covariables; *p* values <0.05 were considered statistically significant.

## 7. Results

### 7.1. General Characteristics of the National Emergency Department Information System Dataset

In total, 9,055,185 cases were registered in the NEDIS dataset during the study period, of which 5,937,569 (65.6%) cases were from EMCs and the remaining 3,117,616 (34.4%) were from local EDs.

### 7.2. Results of Out-of-Hospital Cardiac Arrest Patients Receiving Cardiopulmonary Resuscitation in the Emergency Department

From the study dataset, cases of OHCA patients who received CPR were extracted according to the aforementioned criteria, resulting in 11,493 patients selected for analysis (Figure 1). The EMC group included 8,912 patients, while the local ED group included 2,581 patients. The characteristics of the two groups are summarised in Table 1.

The article "Influence of the Level of Emergency Medical Facility on the Short-Term Treatment Results of Cardiac Arrest: Out-of-Hospital Cardiac Arrest and Interhospital Transfer" was published in 2022. Journal: Emerg Med Int.

There were no statistical differences in age or sex between the groups. The ED mortality was higher in the EMCs than in the local EDs (79.2% vs. 77.2%). Survivors were commonly admitted to the intensive care units in the EMC group, whereas transfer to other hospitals was more common in the local ED group. Additionally, the length of stay in the ED was significantly longer in the EMCs than in the local EDs, which could have contributed to the mortality in the ED rather than death after disposition.

Multivariate logistic regression analysis revealed that the odds for ED mortality were lower with treatment in local EDs than with treatment in EMCs when adjusted for age, sex, and length of stay in the ED. The odds ratio was 0.712 (95% confidence interval (CI): 0.638–0.796).

### 7.3. Treatment Results of Targeted Temperature Management in Emergency Medical Centres Compared between the Direct Visit Group and the Transferred Group

From the study dataset, cases of 1,798 patients who received TTM at the EMCs in hospitals were extracted (Figure 2). Those who were transported directly from the field (direct visit group, *n* = 1,164) and those transferred from other hospitals (transferred group, *n* = 634) were compared. The general characteristics of the two groups are presented in Table 2. Most cases in the direct visit group were transported by National Fire Agency ambulances, which is the predominant prehospital emergency organisation, while other ambulances operated by hospitals or private agencies were mostly utilised for the transferred group. There were no significant differences in age, sex, or severity as represented by the MEWS between the two groups, although there were statistically significant differences in consciousness and systolic blood pressure. The ED disposition and results after admission did not differ significantly between the two groups.

The multivariate regression analysis showed that the odds ratio for overall mortality, including ED mortality and death after admission, was 1.411 (95% CI: 0.809–2.446) in the transferred group when compared to the direct visit group, but without a statistically significant difference (*P* = 0.220).

## 8. Discussion

This study revealed that the immediate outcome of OHCA patients transported to local EDs was not inferior to that of higher-level EMCs. However, a substantial proportion of survivors in the local EDs were transferred to other hospitals, and the outcome of those transferred patients had to be elucidated. Therefore, we evaluated the outcome of TTM in EMCs to compare the treatment results of OHCA survivors between those directly transported to EMCs and those who underwent inter-hospital transfer. Our results showed that there was no significant difference in in-hospital mortality among the patients receiving TTM between the direct visit group and the transferred group. While our study found an overall survival rate of 9.3% in EMCs and 17.9% in local EDs, the national sudden cardiac arrest survey in Korea reported that the rate of survival discharge among OHCA patients was 7.6% in 2016, which was lower than that of our study [15]. This could be because the survey included patients pronounced dead before or upon arrival at the ED, while our study included patients in whom CPR was performed in the ED only.

The article "Influence of the Level of Emergency Medical Facility on the Short-Term Treatment Results of Cardiac Arrest: Out-of-Hospital Cardiac Arrest and Interhospital Transfer" was published in 2022. Journal: Emerg Med Int.

The current international guidelines for CPR suggest the concept of a CAC equipped with sufficient personnel and equipment for comprehensive post-resuscitation care as well as ACLS [16,17]. The CACs can provide a standardised care plan for post-resuscitated patients as well as general care for critically ill patients [18]. The previous studies suggested that CAC should provide access to interventional cardiology facilities, TTM, diagnostic imaging capability, and standardised neuroprognostication [19–21]. There is currently no accreditation or designation program for CACs in Korea, though most EMCs meet the requirements for post-resuscitation management. Therefore, CACs and EMCs can be considered comparable under the current circumstances in Korea.

Although comprehensive and sophisticated care is available in higher-level centres, transporting patients to these centres would require more time than transporting them to nearby EDs. This could result in delayed initiation of ACLS in countries where prehospital ACLS is not universally available. Park et al. reported that longer transport time intervals adversely affected the chances of good neurological recovery in OHCA patients without prehospital ROSC [22]. On the other hand, some reports state that there is no association between transport time and survival to hospital admission [23] or that better neurological outcome is associated with longer rather than very short prehospital time [24]. However, these results were obtained from EMSs, where prehospital ACLS and termination-of-resuscitation are available; hence, only patients with prehospital ROSC are transported to EMCs. Our study results revealed that local EDs had lower mortality at the time of ED disposition, even after adjusting for a shorter length of stay in the local EDs. This finding indicates that local EDs can provide advanced resuscitation for OHCA patients with sufficient quality and better accessibility, resulting in good immediate outcomes.

The article "Influence of the Level of Emergency Medical Facility on the Short-Term Treatment Results of Cardiac Arrest: Out-of-Hospital Cardiac Arrest and Interhospital Transfer" was published in 2022. Journal: Emerg Med Int.

Although the study revealed that local EDs achieved high rates of survival through hospital admission or ED discharge of patients with OHCA, the proportion of patients transferred to other hospitals was as high as 13.4% of all patients treated, which was more than 50% of the ED survivors. Therefore, the outcomes of patients who underwent interhospital transfers had to be elucidated. However, it was not possible to trace the patients to subsequent ED visits because the anonymised dataset did not allow for this process. Therefore, we analysed the data of patients who received TTM in EMCs and compared the treatment outcomes between those who directly visited the EMCs and those who were transferred from other hospitals. The results showed no significant differences in in-hospital mortality between these two groups.

Several studies have demonstrated the impact of interhospital transfers of OHCA patients on treatment outcomes. Cournoyer et al. suggested that it could be advantageous to redirect OHCA patients to PCI-capable centres if the resulting expected delay was <14 min [25]. A study on long-term outcomes of OHCA care showed that both early interfacility transfer to a cardiac arrest receiving centre and direct transport to a cardiac arrest receiving centre from the scene are independently associated with reduced mortality [5]. A single-centre study conducted in Korea found that the prognosis of OHCA patients did not differ between those directly transported from the field and those transferred from other hospitals after ROSC [8]. Our results confirmed the findings of these studies at a national level by utilising a population-based database on emergency care usage.

This study has several limitations. First, it utilised the dataset on the use of general EDs and it was not specifically designed for studies on cardiac arrests. Therefore, the OHCA cases had to be extracted based on the clinical data and clues such as initial vital signs and insurance claim code of CPR. Similarly, because the cases transferred after ROSC were not explicitly defined, we extracted TTM cases to represent postresuscitation management. It should be noted that not all patients who received TTM had postcardiac arrest syndrome, and some patients with brain injury or in-hospital cardiac arrest might have been included. Second, prehospital parameters, such as prehospital time, initial arrest rhythm, or bystander CPR, were not considered because the NEDIS database did not contain these prehospital variables. However, limitations such as these are common in studies based on preexisting big data at the national level, such as insurance claim data [1, 26]. The value of this study is that it investigated the association between the level of the emergency medical facilities and treatment results of OHCA at a national level, which has rarely been reported to date.

The article "Influence of the Level of Emergency Medical Facility on the Short-Term Treatment Results of Cardiac Arrest: Out-of-Hospital Cardiac Arrest and Interhospital Transfer" was published in 2022. Journal: Emerg Med Int.

## 9. Conclusions

The immediate outcome of OHCA patients who were transported to local EDs was not inferior to that of higher-level EMCs. Therefore, it would be acceptable to transport OHCA patients to the nearest emergency facilities, including local EDs, especially in areas where the capacity for prehospital ACLS is limited.

## Figures and Tables

**Figure 1:** Flow diagram illustrating included and excluded cases of out-hospital cardiac arrest. NEDIS: national emergency department information system; CPR: cardiopulmonary resuscitation; ED: emergency department; SBP: systolic blood pressure; EMC: emergency medical center.

**Figure 2:** Flow diagram illustrating included and excluded cases who received therapeutic hypothermia. NEDIS: national emergency department information system; TTM: targeted temperature management; ED: emergency department.

**Table 1:** Characteristics of patients arrived in out-hospital cardiac arrest and received cardiopulmonary resuscitation in the emergency medical institutions. Values are presented in counts and percentages in parentheses.

	EMC group	Local ED group	*p* value
	(*n* = 8,912)	(*n* = 2,581)	
Number of facilities registered in November 2019	162	240	
Gender (male) (n, %)	5,605 (62.9)	1,617 (62.7)	0.840
*Age (years)*			0.223
15∼24	61 (0.7)	19 (0.7)	
25∼44	451 (5.1)	115 (4.5)	
45∼64	2,323 (26.1)	627 (24.3)	
65∼74	3,122 (35.0)	927 (35.9)	
75 or above	2,955 (33.2)	893 (34.6)	
*ED disposition*			<0.001
Death	7,052 (79.2)	1,986 (77.2)	
Admission to ICU	1,444 (16.2)	209 (8.1)	
Admission to ward	33 (0.4)	17 (0.7)	
Discharge	16 (0.2)	14 (0.5)	
Transfer to another hospital	356 (4.0)	345 (13.4)	
Others	7 (0.1)	3 (0.1)	
Survival in ED (*n*, %)	1,856 (20.8)	594 (23.0)	0.018
*Outcome after hospitalization*			0.001
Death	1,024 (70.7)	132 (66.0)	
Discharge	199 (13.7)	43 (21.5)	
Transfer to another hospital	209 (14.4)	19 (9.5)	
Others	16 (1.1)	6 (3.0)	
Overall survival (n, %)	830 (9.3)	462 (17.9)	<0.001
EDLOS (hours)	145.5 ± 282.4	87.4 ± 111.7	<0.001
Hospital LOS (days)	10.5 ± 19.6	6.6 ± 11.3	<0.001

EMC: emergency medical center; ED: emergency department; ICU: intensive care unit; EDLOS: emergency department length of stay; LOS: length of stay.

The article "Influence of the Level of Emergency Medical Facility on the Short-Term Treatment Results of Cardiac Arrest: Out-of-Hospital Cardiac Arrest and Interhospital Transfer" was published in 2022. Journal: Emerg Med Int.

**Table 2:** Characteristics of patients who received therapeutic hypothermia in the emergency medical centers, either in the emergency departments or after hospitalization. Those who were transported directly and those who were transferred from other hospitals were compared. Values are reported in counts and percentages in parentheses.

	Direct group	Transferred group	*p* value
	*n* = 1,164	*n* = 634	
Gender (male) (n, %)	807 (69.3)	408 (64.4)	0.036
*Age (years)*			0.025
15∼24	25 (2.1)	15 (2.4)	
25∼44	148 (12.7)	87 (13.7)	
45∼64	499 (42.9)	233 (36.8)	
65∼74	364 (31.3)	200 (31.5)	
75 or above	128 (11.0)	99 (15.6)	
*Mode of transport*			<0.001
NFA ambulance	1,092 (93.8)	73 (11.5)	
Other ambulances	19 (1.6)	509 (80.3)	
Air transportation	4 (0.3)	30 (4.7)	
Other transportation	49 (4.2)	22 (3.5)	
*AVPU scale*			<0.001
Verbal	116 (10.0)	52 (8.2)	
Pain	289 (24.8)	260 (41.0)	
Unresponsive	759 (65.2)	322 (50.8)	
Systolic blood pressure (mmHg)	135.3 ± 45.9	125.2 ± 40.4	<0.001
Heart rate (beats per minute)	95.0 ± 29.8	97.6 ± 26.8	0.109
Respiratory rate (breaths per minute)	20.0 ± 5.7	20.2 ± 5.8	0.617
Body temperature (°C)	36.1 ± 1.2	36.2 ± 1.4	0.613
MEWS	5.6 ± 2.3	5.6 ± 2.2	0.781
*ED disposition*			0.531
Death	25 (2.1)	13 (2.1)	
Discharge	2 (0.2)	0 (0.0)	
Admission to ICU	1106 (95.0)	597 (94.2)	
Transfer to other hospital	7 (0.6)	7 (1.1)	
Admission to ward	24 (2.1)	17 (2.7)	
Survival in ED	1,139 (97.9)	621 (97.9)	1.000
*Treatment outcome after hospitalization*			0.103
Death	448 (39.8)	247 (40.4)	
Discharge	354 (31.5)	161 (26.3)	
Transfer to another hospital	310 (27.6)	199 (32.5)	
Hopeless discharge	1 (0.1)	0 (0.0)	
Others	12 (1.1)	5 (0.8)	
Overall survival rate	690 (59.3)	374 (59.0)	0.945

EMC: emergency medical center; NFA: national fire agency; ED: emergency department; MEWS: modified emergency warning score; ICU: intensive care unit.

## Data Availability

The data that support the findings of this study are available from the National Emergency Medical Center of the Republic of Korea, but restrictions apply to the availability of these data, which were used under license for the current study and thus are not publicly available.
